This article has been retracted.

# New Diagnosis and Therapy Model for Ischemic-Type Biliary Lesions following Liver Transplantation—A Retrospective Cohort Study

**DOI:** 10.1371/journal.pone.0105795

**Published:** 2014-09-05

**Authors:** Ying-cai Zhang, En-ze Qu, Jie Ren, Qi Zhang, Rong-qin Zheng, Yang Yang, Gui-hua Chen

**Affiliations:** 1 Department of Liver Transplantation, Third Affiliated Hospital of Sun Yat-Sen University, Guangzhou, China; 2 Department of Medical Ultrasonics, Third Affiliated Hospital of Sun Yat-Sen University, Guangzhou, China; 3 Guangdong Provincial Key Laboratory of Liver Disease, Guangzhou, China; University of Pisa, Italy

## Abstract

Ischemic-type biliary lesions (ITBLs) are a major cause of graft loss and mortality after orthotopic liver transplantation (OLT). Impaired blood supply to the bile ducts may cause focal or extensive damage, resulting in intra- or extrahepatic bile duct strictures or dilatations that can be detected by ultrasonography, computed tomography, magnetic resonance cholangiopancreatography, and cholangiography. However, the radiographic changes occur at an advanced stage, after the optimal period for therapeutic intervention. Endoscopic retrograde cholangio-pancreatography (ERCP) and percutaneous transhepatic cholangiodrainage (PTCD) are the gold standard methods of detecting ITBLs, but these procedures cannot be used for continuous monitoring. Traditional methods of follow-up and diagnosis result in delayed diagnosis and treatment of ITBLs. Our center has used the early diagnosis and intervention model (EDIM) for the diagnosis and treatment of ITBLs since February 2008. This model mainly involves preventive medication to protect the epithelial cellular membrane of the bile ducts, regular testing of liver function, and weekly monitor of contrast-enhanced ultrasonography (CEUS) to detect ischemic changes to the bile ducts. If the liver enzyme levels become abnormal or CEUS shows low or no enhancement of the wall of the hilar bile duct during the arterial phase, early ERCP and PTCD are performed to confirm the diagnosis and to maintain biliary drainage. Compared with patients treated by the traditional model used prior to February 2008, patients in the EDIM group had a lower incidence of biliary tract infection (28.6% vs. 48.6%, *P* = 0.04), longer survival time of liver grafts (24±9.6 months vs. 17±12.3 months, *P* = 0.02), and better outcomes after treatment of ITBLs.

## Introduction

Advances in organ preservation techniques, immunosuppressive regimens, and surgical techniques have resulted in reduced rates of infection, acute rejection and vascular complications after orthotopic liver transplantation (OLT). However, ischemic-type biliary lesions (ITBLs) are still one of the most serious complications after OLT, with a usual reported incidence of 5–15% [1]–[7], and an incidence of up to 26% in some studies [8], [9]. OLT recipients have a graft loss rate of up to 46% after 2 years, and ITBLs are one of the major causes of graft loss requiring re-transplantation [10]. The traditional methods of diagnosing ITBLs depend mainly on interventional imaging techniques, such as magnetic resonance cholangiopancreatography (MRCP), endoscopic retrograde cholangio-pancreatography (ERCP) or percutaneous transhepatic cholangiodrainage (PTCD). However, these methods are unable to provide early diagnosis and therapy, and it would be beneficial to develop a method of early prediction and diagnosis of ITBLs. This study aimed to evaluate the efficacy of the early diagnosis and intervention model (EDIM), which has been used in our department for the diagnosis and treatment of ITBLs after OLT since February 2008.

## Materials and Methods

### Patients

From October 2003 to June 2012, 594 patients underwent OLT at the Liver Transplantation Center, Third Affiliated Hospital of Sun Yat-sen University. Based on the different models used for the diagnosis and therapy of ITBLs, patients who were diagnosed with ITBLs after OLT from October 2003 to January 2008 (first period) were allocated to the control group, and patients who were diagnosed with ITBLs from February 2008 to June 2012 (second period) were allocated to the EDIM group. Table 1 shows the clinical characteristics of patients in the two groups. The control group included 37 patients with ITBLs (32 males, 5 females) with a mean age of 49.7 years (range 26–70 years) at the time of OLT. The EDIM group included 28 patients with ITBLs (25 males, 3 females) with a mean age of 46.6 years (range 29–62 years) at the time of OLT.

**Table 1:** Demographic and clinical characteristics of OLT patients during the two periods.

	First period (n = 290)	Second period (n = 304)	*P* value
**Age** (year)	46.2±13.2	43.4±12.3	0.314
**Gender** (F/M)	53/237	64/240	0.395
**WIT** (minute)	6.3±3.3	6.8±3.6	0.272
**CIT** (hour)	9.2±3.4	8.7±2.9	0.256
**Anhepatic time** (min)	50±6.4	48±5.7	0.381
**Operation time** (hour)	7.1±2.4	6.9±2.1	0.527
**Preservation solution** (UW/Celsior)	221/69	217/87	0.182
**ITBLs patient** (%)	37 (12.8%)	28 (9.2%)	0.167

OLT: orthotopic liver transplantation; WIT: warm ischemia time; CIT: cold ischemia time.

The diagnostic criteria for ITBLs were: (1) focal or extensive damage to the bile ducts, characterized by intra- or extrahepatic strictures, necrosis, and destruction detected by cholangiography; and (2) absence of hepatic artery thrombosis, ABO incompatibility, biliary anastomotic stricture, or other reasons for biliary destruction.

The inclusion criteria for the study were: (1) confirmation of ITBLs by cholangiography; and (2) good compliance with regular follow-up. The exclusion criteria were: (1) death not due to bile duct complications; (2) primary sclerosing cholangitis as the primary disease; and (3) incomplete follow-up.

Routine biochemical testing and US/CEUS were performed by a member of the transplant team on an outpatient basis. The outpatient follow-up visits were usually once a week during the first month after discharge, twice a month during the second and third months and then monthly until the end of the first year, and every 3 or 4 months thereafter; and at any time there was an indication of a potential problem.

All the patients in the EDIM group gave written informed consent. The study was approved by the Ethics Committee of the Third Affiliated Hospital of Sun Yat-Sen University, and followed the STROBE guidelines for reporting of observational studies.

### CEUS apparatus and Methods

CEUS was performed with an An Acuson Sequoia 512 ultrasound machine with a 4V1 convex array probe (1.0–4.0 MHz), using a contrast pulse sequence model with a mechanical index of 0.15–0.21. SoneVue contrast (Bracco, Italy) was diluted in 5 mL of saline to form sulfur hexafluoride microbubbles and was repeatedly injected into a superficial cubital vein (1.5 mL/injection).

### Procedures for the diagnosis and treatment of ITBLs

In the control group, ultrasonography and MRCP were used for the preliminary diagnosis of ITBLs in OLT-recipients who developed cholangitis, jaundice, or liver function abnormality. ERCP or PTCD were performed to confirm the ITBLs diagnosis and maintain the patency of the biliary drainage. Medications were administered as required, and partial hepatectomy and/or choledochojejunostomy were performed in some cases. Re-transplantation was considered only when the above strategies failed (Figure 1).

**Figure 1:** Algorithm for the diagnosis and treatment of ITBLs after OLT in the control group. ERCP, endoscopic retrograde cholangio-pancreatography; ITBLs, ischemic-type biliary lesion; MRCP, magnetic resonance cholangiopancreatography; OLT, orthotopic liver transplantation; PTCD, percutaneous transhepatic cholangiodrainage.

In the EDIM group, OLT-recipients were prophylactically treated with ursodeoxycholic acid, ademetionine and prostaglandin-E after OLT. The serum alanine aminotransferase, total bilirubin and Gamma-glutamyl transpeptidase levels were routinely monitored. CEUS was performed weekly in the early stage after OLT (<3 months). If there was an increase in the Gamma-glutamyl transpeptidase level and CEUS showed no or low enhancement of the wall of the hilar bile duct during the arterial phase, PTCD or ERCP was performed to confirm the diagnosis of ITBLs and maintaini the patency of the biliary drainage at the same time. Re-transplantation was the last option if interventional therapy, partial hepatectomy and/or hepato-enterostomy failed to resolve the ITBLs (Figure 2).

**Figure 2:** Algorithm for the diagnosis and treatment of ITBLs after OLT in the EDIM group. CEUS, contrast-enhanced ultrasonography; EDIM, early diagnosis and intervention mode; ERCP, endoscopic retrograde cholangio-pancreatography; ITBLs, ischemic-type biliary lesion; MRCP, magnetic resonance cholangiopancreatography; OLT, orthotopic liver transplantation; PTCD, percutaneous transhepatic cholangiodrainage.

### Statistical analysis

All statistical analyses were performed using SPSS 15.0 software (SPSS Inc., IL, USA). Continuous variables are presented as the mean ± standard deviations, and categorical variables are presented as percentages. Quantitative variables were compared using the Student's t test or Mann-Whitney U test, and qualitative variables were compared using the χ^2^ test or Fisher's exact test. Survival curves were compared using the nonparametric Log-Rank tests. A *P* value of <0.05 was considered to indicate statistical significance.

## Results

### Postoperative Follow-Up

All patients in the study were followed up until July 2013. The median follow-up period of the 37 patients in the control group was 61.4±11.2 months (range 6–98 months), and of the 28 patients in the EDIM group was 38.4±7.2 months (range 11–57months).

### Diagnosis of ITBLs using CEUS

In patients without ITBLs, the wall of the hilar bile duct was significantly enhanced during the arterial phase (more than the liver parenchyma) (Figure 3). In patients with ITBLs, there was no or low enhancement of the wall of the hilar bile duct during the arterial phase (Figure 4).

**Figure 3:** Ultrasound image of the hilar bile duct in a patient without ITBLs. **B:** Regular ultrasound image showing a thickened hilar bile duct wall with a high echogenicity (arrow) and an obscure lumen. **A:** Arterial stage of CEUS showing high enhancement of the bile duct (arrow) and a clear lumen. CEUS: contrast-enhanced ultrasound; OLT: orthotopic liver transplantation.

**Figure 4:** Ultrasound image of the hilar bile duct in a patient with ITBLs. **B:** Regular ultrasound image showing a thickened hilar bile duct wall with equal echogenicity (arrow) and an obscure lumen. **A:** Arterial stage of CEUS showing low enhancement in the bile duct wall (arrow) and a clear lumen.

### Differences in the Timing of ITBLs Diagnosis and Treatment

The time from OLT to biliary intervention was significantly longer in the control group (105.1±41.9 days) than in the EDIM group (57.6±18.2 days) (*P* = 0.007). ITBLs were diagnosed and treated earlier in the EDIM group than in the control group. In addition, earlier biliary intervention to maintain the patency of the biliary drainage significantly decreased the incidence of biliary infection in the EDIM group compared with the control group (28.6% vs. 48.6%, *P* = 0.04).

### Survival of Transplanted Livers and Hosts

The liver function improved after interventional and/or surgical therapy in 18 patients in the control group and 20 patients in the EDIM group. Repeat transplantation after failure of the above interventions was required in 11 patients in the control group and six patients in the EDIM group. Eight patients in the control group and two patients in the EDIM group died before re-transplantation was performed. The 1- and 3-year graft survival rates were 78.4% and 53.2% in the control, and 92.9% and 78.6% in the EDIM group. The graft survival rate was significantly poorer in the control group than in the EDIM group (*P* = 0.008 Figure 5). The mean time of graft loss was significantly longer in the EDIM group (24±9.6 months, range 11–41 months) than in the control group (17±12.3 months; range 6–44 months) (*P* = 0.02).

**Figure 5:** Survival times of liver grafts in the two groups. The 1- and 3-year graft survival rates were 78.4% and 53.2% in the control group and 92.9% and 78.6% in the EDIM group (*P* = 0.008).

## Discussion

ITBLs after OLT are difficult to diagnose and treat. Currently, the diagnosis of ITBLs after OLT depends mainly on cholangiography during investigations such as MRCP, ERCP and PTCD [5], [6], [10]–[12]. MRCP is a non-invasive investigation that is becoming the first choice for diagnosis of ITBLs [13]–[15]. Borasci et al. reported that MRCP had a sensitivity of 93%, specificity of 92%, positive predictive value of 86%, and negative predictive value of 96% for the the diagnosis of biliary complications after OLT [13]. MRCP can detect tortuosity and deformity of the biliary tree, cholangiectasis of the intrahepatic ducts, accumulation of biliary sludge and destruction of the bile ducts. However, these changes do not occur until the advanced stages of ITBLs, after the optimal period for therapeutic intervention. ERCP and PTCD are currently the gold standard methods for diagnosing ITBLs. However, ERCP and PTCD are both invasive and can cause pancreatitis or bleeding [16], [17], and are therefore not suitable for early monitoring and diagnosis of ITBLs after OLT. It is important to develop an easy and a non-invasive method for early diagnosis of ITBLs.

CEUS is an ultrasonic examination method that increases the difference in echogenicity, between blood and tissue by injection of ultrasonic contrast agent into the blood. Animal and clinical experiments have shown that the microbubble-to-tissue signal ratio after injection of ultrasonic contrast agent can be used to observe flow that may be difficult to detect on color Doppler ultrasonography, such as in deep vessels or in low-velocity vessels such as the microcirculation [18], [19]. CEUS is therefore an important investigation for the diagnosis of hepatic artery and portal vein complications after OLT, and reduces the need for more invasive investigations such as angiography [18], [20]–[23]. However, few studies have focused on using CEUS for the diagnosis of biliary complications such as ITBLs after OLT. The blood supply of the bile ducts depends entirely on the arterial peribiliary plexus, which is perfused by the gastroduodenal and hepatic arteries. Damage to the peribiliary vascular plexus may cause microcirculatory changes, resulting in necrosis, fibrosis, and stenosis of the biliary tract [9], [24]–[26]. SonoVue, the ultrasonic contrast agent used for CEUS, differs from the contrast used for computed tomography and magnetic resonance imaging, SonoVue is a blood pool agent that gives a more reliable depiction of tissue microcirculation because the microbubbles are not small enough to pass through the microvascular endothelial gap [27]. Use of CEUS to monitor microcirculatory changes to the peribiliary vascular plexus after OLT may enable early diagnosis of ITBLs.

Our previous study showed a significant difference in the enhancement of the hilar bile duct on CEUS between patients with and without ITBLs. During the arterial phase of CEUS, there was no or low enhancement of the wall of the hilar bile duct in patients with ITBLs. In patients without ITBLs, there was more enhancement of the hilar bile duct walls than of the hepatic parenchyma in the arterial phase, followed by similar or lower enhancement of the hilar bile duct walls compared with the hepatic parenchyma in the portal venous and late phases [28]. The CEUS finding reflects the extent of damage to the peribiliary vascular plexus, and the extent of decreased perfusion to the bile duct. These changes help to diagnose ITBLs before the development of morphological changes to the bile duct. Another study by our group showed that CEUS had a sensitivity of 64.6%, specificity of 88.9%, and accuracy of 75.0% for diagnosing ITBLs [29]. It therefore seems feasible to diagnose ITBLs during the period of functional changes to the bile duct.

This study also evaluated a new model for the treatment of for ITBLs. Previously, medication, interventional and other therapies were administered after ITBLs was diagnosed by ERCP or PTCD. It usually takes 3–5 months to confirm the diagnosis of ITBLs using these methods. Unfortunately, delayed diagnosis is a major risk factor for the irreversible biliary damage. Bile salt retention is a major risk factor for the hepatocellular and biliary injury after OLT [1]. Hertl et al. reported that damage to the intrahepatic biliary duct after OLT was significantly increased when pig livers were flushed with saline containing hydrophobic bile salts compared with being flushed with saline alone [30]. Hoekstra et al. found that intrahepatic bile salt retention was an important mechanism of graft damage after OLT in transgenic mice [31]. In humans, damage to the bile duct is associated with toxic bile, characterized by a high cholate/phospholipid ratio [32]. Salt retention also results in bacterial growth and an increased risk of biliary tract infection. Considering the findings of these previous studies, we believe that it is important to maintain the patency of the biliary tree to prevent salt retention and protect the bile duct epithelium by performing early biliary intervention (PTCD or ERCP). In February 2008, we started to administer oral ursodeoxycholic acid and ademetionine immediately after OLT to prevent bile deposition and gallstone formation, and intravenous prostaglandin-E to improve the microcirculation of the peribiliary vascular plexus and to reduce damage to the biliary epithelial cells. When the CEUS findings indicated ITBLs, PTCD or ERCP were routinely performed to confirm the diagnosis and maintain biliary drainage. The EDIM achieved early diagnosis and treatment of ITBLs, resulting in reduced damage to the bile ducts, a lower incidence of biliary tract infection, longer survival time of liver grafts, and reduced graft loss compared with traditional treatment methods.

In summary, the traditional methods of follow-up and diagnosis result in delayed diagnosis and treatment of ITBLs after OLT compared with regular monitoring with CEUS. Prophylactic medications, earlier detection, and earlier intervention may lead to improved outcomes in patients with ITBLs.
